# Calmodulin-binding transcription activator (CAMTA) genes family: Genome-wide survey and phylogenetic analysis in flax (*Linum usitatissimum*)

**DOI:** 10.1371/journal.pone.0236454

**Published:** 2020-07-23

**Authors:** Essa Ali, Mohammad Ammar Raza, Ming Cai, Nazim Hussain, Ahmad Naeem Shahzad, Mubshar Hussain, Murtaza Ali, Syed Asad Hussain Bukhari, Peilong Sun

**Affiliations:** 1 Department of Food Science and Technology, Zhejiang University of Technology, Hangzhou, Zhejiang, China; 2 School of Food Science and Biotechnology, Zhejiang Gongshang University, Hangzhou, Zhejiang, China; 3 College of Agriculture and Biotechnology, Zhejiang University, Hangzhou, China; 4 Department of Agronomy, Bahauddin Zakariya University, Multan, Pakistan; 5 Department of Basic Science & Humanities, University of Engineering and Technology, Mardan, Pakistan; Harran University, TURKEY

## Abstract

Flax (*Linum usitatissimum*) is a member of family linaceae with annual growth habit. It is included among those crops which were domesticated very early and has been used in development related studies as a model plant. In plants, Calmodulin-binding transcription activators (CAMTAs) comprise a unique set of Calmodulin-binding proteins. To elucidate the transport mechanism of secondary metabolites in flax, a genome-based study on these transporters was performed. The current investigation identified nine CAMTAs proteins, classified into three categories during phylogenetic analysis. Each group had significant evolutionary role as illustrated by the conservation of gene structures, protein domains and motif organizations over the distinctive phylogenetic classes. GO annotation suggested a link to sequence-specific DNA and protein binding, response to low temperature and transcription regulation by RNA polymerase II. The existence of different hormonal and stress responsive *cis-*regulatory elements in promotor region may directly correlate with the variation of their transcripts. MicroRNA target analysis revealed that various groups of miRNA families targeted the *LuCAMTAs* genes. Identification of *CAMTA* genes, miRNA studies and phylogenetic analysis may open avenues to uncover the underlying functional mechanism of this important family of genes in flax.

## Introduction

The divalent ions of calcium (Ca^2+^) play a key role as core transducers and regulators in response to environmental stimuli and processes related to development of plants [1]. Ca^2+^ signals are decoded into appropriate physiological responses and transmitted to their different loading statuses [2, 3]. The known classes of Ca^2+^ sensors in plants include calcium dependent protein kinases (CDPKs), calcineurin B-like proteins (CBLs) and calmodulins (CaMs) [4]. Among the reported plant sensors, Calmodulins (CaMs) are the well-studied Ca^2+^ binding proteins that physically attach to a huge number of target proteins such as phosphatases, protein kinases, metabolic enzymes, transcription factors, ion channels, molecular motors and transporters [2, 5]. Calmodulins-regulated Transcription factors (TFs) are important in these processes and about ninety such TFs are reported as CaM-binding proteins (CBPs) [3, 6–8]. Among these TFs, CAMTAs comprise the newest and unique set of CaM-binding proteins (CBPs) in plants [9]. The tobacco early ethylene-responsive gene (NtER1) was the very first identified *CAMTA* gene in tobacco which is known to be involved in senescence and death of plants. In addition, many eukaryotes have been identified to be equipped with CAMTA transporters including *Arabidopsis thaliana* [9], *oryza sativa* [10], *Vitis vinifera* [11], *Brassica napus* [12], *Lycopersicum esculantum* [13], *Medicago truncatula* [14], *Citrus sinensis* [15], *Populus trichocarpa* [16], *Nicotiana tabacum* [17], *Musa acuminata* [18], *Phaseolus vulgaris* [19], *Zea mays* [20], *Solanum lycopersicum* [21], *Fragaria ananassa* [22], and *Glycine max* [23]. The CAMTA-encoded proteins of plants are characterized with the presence of four functional domains known as IPT/TIG (transcription factor immunoglobulin), IQ motifs (calmodulin-binding), CG-1 (a DNA-binding domain specific to sequence), and ankyrin (ANK) repeats [24–27]. The binding site for CAMTAs are present in downstream promoter regions of the target genes and designated as A/C/G)CGCG(T/C/G) or (A/C)CGTGT, which helps to regulates its expression [10, 28]. Six CAMTA transporters named as AtCAMTA1 to AtCAMTA6 have been identified in Arabidopsis. These AtCAMTAs are involved in biotic, abiotic and hormonal regulations [28–31]. For instance, AtCAMTA1 and AtCAMTA3 play roles against freezing and drought stress as well as regulation of auxin and salicylic acid in plants [31–35]. AtCAMTA6 support the plants against salt stress, while AtCAMTA4 performs pivotal role in defense responses of plants against *Puccinia triticina* and low temperature stress [36, 37].

Flax (*Linum usitatissimum*), an annual plant of family Linaceae, is considered among the very first domesticated crops in the world. It has been utilized as a model species to investigate the development related processes in plants [38]. Seeds of flax have bulk amounts of essential fatty acids i.e. omega-3 fatty acids [39], which mitigate the inflammatory reactions and reduce the risk of cardiovascular diseases [40]. Moreover, other polyunsaturated fatty acids (PUFAs), present in flaxseeds, may protect the retina from harmful effects of diabetes mellitus type 2 [41]. Flaxseeds also possess lignans, which act as antioxidant due to their ability of scavenging free radicals [42]. Additionally, lignans perform pivotal roles to inhibit breast, lung and colorectal cancer [43–45]. Flaxseed oil also supports kidneys against the detrimental effects of heavy metals [46]. Mucilage of raw flaxseed is used in dairy products as a stabilizing agent [47]. Bio-active compounds, present in flax, may control inflammation, metabolic disorders, constipation, hypertension, obesity and lipid level [48, 49]. As the genome of flax has been sequenced [50], a number of studies has been conducted revealing the role of several flax genes under environmental stresses and hormonal signaling [51–55]. Despite of being an important crop, so far no report has been published regarding CAMTA transporters in flax (*Linum usitatissimum*).

The current study was carried out to understand the diversity and evolutionary conservation of *CAMTA* gene family in flax. Multiple approaches were employed for detailed study of each member of CAMTA gene family, along with the investigation on physiological characteristics of corresponding proteins.

## Methodology

### Identification of CAMTAs in flax genome

The Arabidopsis information resource (http://www.arabidopsis.org/) database was accessed to download the sequences of six CAMTA family members from *Arabidopsis thaliana* [56]. BLASTP (E-value was ≤ 1e^-7^) search was made against the genome of flax in Phytozome database (v. 12.1) (http://www.phytozome.net/) [57] using Arabidopsis CAMTA proteins as queries. Pfam (http://pfam.xfam.org/) [58], SMART (http://smart.embl-heidelberg.de/smart/batch.pl) [59] and conserved domain database (http://www.ncbi.nlm.nih.gov/Structure/cdd/wrpsb.cgi/) [60] were used to collect, screen out and filter non-redundant CAMTA sequences for conserved CAMTA domains. The sequences were evaluated against the potential features of the CAMTA transporters such as the presence of IQ (PF00612), ANK (PF12796), TIG (PF01833) and CG-1 (PF03859) domains. The undesired gene sequences were eliminated manually. ProtParam (http://www.expasy.org/tools/protparam.html) was employed to estimate the physical attributes of CAMTA transporters like molecular weight, isoelectric point, protein size, instability index, aliphatic index, and GRAVY [61]. Further, the subcellular localization of CAMTA proteins were predicted by using the CELLO version 2.5 (http://cello.life.nctu.edu.tw/) [62] and WoLF PSORT (http://www.genscript.com/wolf-psort.html) [63].

### Phylogenetic analysis of flax CAMTA proteins

CAMTA protein sequences were aligned in Arabidopsis and flax by using the Clustal W function of MEGA 7.0. The MEGA 7.0 software was used to construct the phylogenetic tree [64], applying the Maximum Likelihood algorithm with 1000 bootstraps replicates. The amino acid substitution model was kept at an equal input model having uniform rates among sites and partial deletion (95% site coverage as cut off) was use for missing data and gaps. The sequence of CAMTA protein of *Arabidopsis thaliana* was used as the control. The family members of LuCAMTAs were named according to the similarity of sequence and its arrangement in the phylogenetic tree.

### Gene structure and motif composition analysis of CAMTAs in flax

The coding DNA sequences of flax *CAMTAs* were run against their corresponding genomic sequences to find out the gene structure by using Gene Structure Display Server (GSDS: http://gsds.cbi.pku.edu.cn) [65]. Moreover, the conserved motifs in flax CAMTA proteins were identified using Multiple Expectation Maximization for Motif Elicitation program (MEME) (http://meme-suite.org/tools/meme) [66]. The parameters were kept as follows; the maximum number of motifs were set at 12, Motif Width was in range from 6 to 50, Site Distribution: zero or one occurrence.

### Analysis of *cis*- regulatory elements in the flax *CAMTA* promoters

Promotor region 1kb upstream for *LuCAMTA* genomic DNA was retrieved from Phytozome database [57]. The sequences obtained were then individually analyzed by submitting to PlantCARE database (http://bioinformatics.psb.ugent.be/webtools/plantcare/html/) [67] with default limitations to identify the key *cis*-regulatory elements with respect to stress and hormonal response.

### Gene ontology annotation and identification of miRNA target sites

Blast2GO software (https://www.blast2go.com/) was employed for gene ontology of the LuCAMTA family members [68]. Biological processes, BP; cellular components, CC and molecular functions, MF; were set as the basis for gene ontology (GO) annotation. The miRNA sequences of flax were retrieved from the miRBase database (http://mirbase.org/) [69], and online repository sRNAanno (http://www.plantsrnas.org/) [70]. The target genes of miRNAs were predicted by employing psRNATarget (http://plantgrn.noble.org/psRNATarget/analysis/) [71].

## Results

### Identification of the members of *CAMTA* gene family in flax

For a comprehensive overview of the *CAMTA* gene family, flax genome was searched against identified six *CAMTA* genes of *A*. *thaliana* as queries in BLAST search of the Phytozome database. All non-redundant putative gene sequences were extracted from the database. SMART, CDD and PFAM databases were used for sequence analysis to confirm the existence of CAMTA-specific conserved domains i.e. IQ: calmodulin-binding IQ motifs, ANK: ankyrin repeats, IPT/TIG: Ig-like, transcription factor immunoglobulin, and CG-1: DNA-binding domain. Nine genes were finally selected and named as *LuCAMTA1–9* for *L*. *usitatissimum* based on their position in relation to *A*. *thaliana* in the phylogenetic tree. The detailed physiological characteristics of the selected LuCAMTA proteins, such as isoelectric point (pI), molecular weight, length, Instability index, Aliphatic index, predicted subcellular locations and GRAVY are presented in Table 1. The size of translated proteins ranged between 850 (LuCAMTA9) and 1103 (LuCAMTA1) amino acids. The molecular weight (M.wt) of the proteins ranged from 94.32 (LuCAMTA9) to 123.63 kDa (LuCAMTA1), and the pI values varied between 6.02 (LuCAMTA1) and 8.26 (LuCAMTA3). The Instability index lies in the range of 39.12 to 46.6 for LuCAMTA4 and LuCAMTA9, respectively. Aliphatic index and GRAVY were found lowest (75.67 and -0.621) to highest (86.12 and -0.357) for LuCAMTA3 and LuCAMTA8, respectively. Subcellular localization of the various CAMTA

**Table 1:** List of identified *CAMTA* genes in flax and their properties.

Groups	Gene names	Accession no	Scaffold			Protein Size	M.wt	Pi	Instability index	Aliphatic index	GRAVY	Localization
			Location	Start	End							
Group-I	LuCAMTA 1	Lus10003405	644	19853	26672	1103	123.63	6.02	46.08	79.66	-0.465	Nuc^a^, Cp^b^
	LuCAMTA 2	Lus10024044	353	205608	211044	959	107.68	7.61	43.59	75.77	-0.564	Nuc^a,b^
	LuCAMTA 3	Lus10041704	272	1360328	1365986	973	109.95	8.26	42.46	75.67	-0.621	Nuc^a,b^
Group-II	LuCAMTA 4	Lus10003119	1847	2666	6412	900	100.93	6.05	39.12	78.46	-0.512	Nuc^a,b^,
	LuCAMTA 5	Lus10011352	744	129430	138462	1076	120.83	6.31	43.01	83.38	-0.363	Nuc^a^, Pm^a,b^
Group-III	LuCAMTA 6	Lus10016873	153	370083	375177	901	100.91	6.42	41.51	80.77	-0.417	Nuc^a,b^
	LuCAMTA 7	Lus10037738	196	1328645	1333781	963	107.72	6.78	42.31	86.12	-0.357	Nuc^a,b^
	LuCAMTA 8	Lus10036455	57	712304	719459	963	107.72	6.78	42.31	86.12	-0.357	Nuc^a,b^
	LuCAMTA 9	Lus10041126	280	1067255	1072213	850	949.32	7.39	46.6	80.33	-0.434	Nuc^a,b^

pI, Isoelectric point; M.wt, Molecular weight; Cp, Chloroplast; Pm, Plasma membrane; Nuc, Nucleus. aLocalization predicted by CELLO v.2.5. bLocalization predicted by pSORT.

The protein sequences were reanalyzed for subcellular localization with CELLO v. 2.5 (http://cello.life.nctu.edu.tw/) to revalidate the outcomes of pSORT. According to the predicted results majority of the CAMTA proteins were localized in the nucleus. However, LuCAMTA1 and LuCAMTA5 were also present in chloroplast and plasma membrane, respectively.

### Phylogenetic analysis of Flax CAMTA protein

To explain the evolutionary conservation of CAMTA proteins in flax, a phylogenetic tree among six CAMTA proteins from *Arabidopsis* and nine CAMTA proteins from flax was constructed. Based on phylogenetic tree, the LuCAMTA protein from flax clustered with AtCAMTAs into three groups (Fig 1A) i.e. I, II and III, which agrees with what has been reported for *Arabidopsis* CAMTAs. The CAMTA proteins of flax were named based on their relationship with known AtCAMTAs. Further, construction of individual phylogenetic tree based on aligned flax CAMTA proteins (Fig 1B), revealed alike cluster arrangements. The size of every LuCAMTA group was different from one another. Group I, II and II contained 03, 02 and 04 members, respectively.

**Fig 1:** Phylogenetic trees of *Arabidopsis thaliana* and flax CAMTA proteins. Combined (A) and flax alone (B). Phylogenetic trees were made with maximum likelihood by using the Neighbor joining model and MEGA 7.0 software. Different colors of branches represent different groups.

### Analysis of *CAMTA* gene structures in flax

For comprehensive understanding of evolution of *CAMTA* genes in flax, their structural analysis was performed. GSDS software was used to make a comparison between coding DNA sequences; CDSs, and their corresponding genomic sequences (Fig 2). Intron number of the genes ranged from 9 to 12 with a little variation in different groups. The *CAMTA* genes, for example, in group II were disrupted by 9–11 introns, while in group I and III they were disrupted by 9–12 introns. The intron phases were 0, 1, and 2.

**Fig 2:** Gene structural analysis of *LuCAMTA*. Exons are presented by red filled boxes and introns are presented by blue lines. The number above introns are representing intron phases. The relative sizes of the intron and exon regions can be deduced from the scale provided in kilobase pair (kb).

### Analysis of motif composition of CAMTA proteins in flax

MEME online database was used for the analysis of conserved motifs of LuCAMTAs encoding proteins. Ten conserved regulatory motifs were identified in *LuCAMTAs* genes and were named as motifs 1–10. The schematic presentation of the motifs identified among different subfamilies is given in Fig 3.

**Fig 3:** Analysis of conserved motifs of nine LuCAMTA proteins. Number assigned by MEME is mentioned on each motif. The figure is recreated with software, DOG 2.0: illustrator of protein domain structures.

Out of 10 identified motifs, 7 and 10 are unknown and are not associated with any known domains in pfam. The functionality of these unknown motifs awaits further experimental proof. Motif 2, 5 and 6 are related to CG-1 domain, while motif 3 correlates with ANK domain and consist of 50 amino acid residues. Motif 1 and 8 are linked to IQ domain, while motif 9 represents IPT/TIG domain. The sequence logo of all the identified motifs are presented in Fig 4.

**Fig 4:** Analysis of the sequence logo of all the identified motifs of LuCAMTAs.

### Prediction of *cis-* regulatory elements in the *LuCAMTA* promoters

To understand the transcriptional and hormonal regulation in response to stress, PlantCARE database was accessed for the prediction of *cis-* regulatory elements in 1000 bp upstream promotor region of *LuCAMTA*. The *LuCAMTAs* promoters have various *cis*- regulatory elements that are believed to be involved in stress responses and hormonal regulations (Fig 5). In this study, the elements identified in response to various stresses include ARF (anaerobic induction), LTR (responsive to low temperature), MBS (responsive to drought) and G-box (responsive to light). During the analysis of promoters, the elements responsive to hormones were also identified. They include abscisic acid-responsive elements (ABRE) and salicylic acid-responsive elements (TCA-element). LuCMATA1, LuCMATA5 and LuCMATA9 have the maximum number of *cis* regulatory elements in their promotor regions.

**Fig 5:** Analysis of the putative promoters of *LuCAMTA* genes for *cis*- regulatory elements by PlantCARE. Bar diagram presents various elements responsive to hormones and stress. Different colors represent the abundance of distinct regulatory elements on each of the promoter.

### Gene ontology annotation of *LuCAMTA* genes in flax

Gene Ontology database was accessed to analyze the functional classification of proteins of the *CAMTA* genes family of flax. The outcomes of the analysis revealed that LuCAMTA proteins were involved in different functions like molecular functions (MF), biological processes (BP), cellular structural components (CC). For cellular structural component (CC), LuCAMTAs were involved in the intracellular and cellular anatomical entity. The genes, specific to molecular functions (MF), were involved in sequence-specific DNA binding activities, while in biological processes (BP), the genes were responsible for response to stimuli and regulation of biological and metabolic processes (Fig 6). Table 2 presents the functions of different *LuCAMTA* genes. Regarding MF, the genes were annotated for protein binding (GO:0005515), DNA binding (GO:0003677), and sequence-specific DNA binding (GO:0043565). In BP, the genes were involved in response to low temperature stress (GO:0009409) and up-regulation of transcription by RNA polymerase II (GO:0045944). Regarding CC, nucleus (GO:0005634), intracellular (GO:0005622) and cellular anatomical entity (GO:0110165) were found in GO functional annotation.

**Fig 6:** GO functional annotation for the flax *CAMTA* genes. Cellular components, molecular functions and biological processes are detected for LuCAMTAs. The different colors represent the proportions of various GO functions.

**Table 2:** Gene Ontology (GO) terms annotation of CAMTA genes in Flaxseed.

Protein Names	Biological Process IDs	Biological Process Names	Molecular Function IDs	Molecular Function Names	Cellular Component IDs	Cellular Component Names
**LuCAMTA01**	P:GO:0045944	P:positive regulation of transcription by RNA polymerase II	F:GO:0043565	F:sequence-specific DNA binding	C:GO:0005634	C:nucleus
			F:GO:0005515	F:protein binding		
			F:GO:0003677	F:DNA binding		
**LuCAMTA02**	P:GO:0045944	P:positive regulation of transcription by RNA polymerase II	F:GO:0005515	F:protein binding	C:GO:0005634	C:nucleus
			F:GO:0003677	F:DNA binding		
**LuCAMTA03**	P:GO:0045944	P:positive regulation of transcription by RNA polymerase II	F:GO:0005515	F:protein binding	C:GO:0005634	C:nucleus
			F:GO:0003677	F:DNA binding		
**LuCAMTA04**	P:GO:0045944	P:positive regulation of transcription by RNA polymerase II	F:GO:0005515	F:protein binding	C:GO:0005622	C:intracellular
			F:GO:0003677	F:DNA binding	C:GO:0110165	C:cellular anatomical entity
**LuCAMTA05**	P:GO:0045944	P:positive regulation of transcription by RNA polymerase II	F:GO:0005515	F:protein binding	C:GO:0005622	C:intracellular
			F:GO:0003677	F:DNA binding	C:GO:0110165	C:cellular anatomical entity
**LuCAMTA06**	P:GO:0045944	P:positive regulation of transcription by RNA polymerase II	F:GO:0043565	F:sequence-specific DNA binding	C:GO:0005634	C:nucleus
			F:GO:0003677	F:DNA binding		
			F:GO:0005515	F:protein binding		
**LuCAMTA07**	P:GO:0045944	P:positive regulation of transcription by RNA polymerase II	F:GO:0043565	F:sequence-specific DNA binding	C:GO:0005634	C:nucleus
			F:GO:0003677	F:DNA binding		
			F:GO:0005515	F:protein binding		
**LuCAMTA08**	P:GO:0009409	P:response to cold	F:GO:0003677	F:DNA binding	C:GO:0005634	C:nucleus
			F:GO:0005515	F:protein binding		
**LuCAMTA09**	P:GO:0045944	P:positive regulation of transcription by RNA polymerase II	F:GO:0003677	F:DNA binding	C:GO:0005634	C:nucleus
			F:GO:0005515	F:protein binding		

### MicroRNAs (miRNA), targeting Lu*CAMTA* genes

MicroRNAs (miRNAs) play a pivotal role in controlling the expression pattern of transcription factors. In the current study, potential miRNAs were searched for a set of nine identified LuCAMTA transcripts by accessing the psRNATarget (plant small-RNA target analysis server). Results demonstrate that all *LuCAMTA* genes, except *LuCAMTA9*, were the targets of eleven different categories of miRNAs (Table 3). These miRNAs are related to various miRNA families such as miRN30, miRN9, miR2275, miR164, miR159, miR164, miRN15, miR395, miR156, miRN28 and miR164. Predicted regulatory mechanism of miRNAs revealed that a single miRNA can target multiple *LuCAMTA* genes (Table 3). For instance, Lus-miR156 targets three *LuCAMTAs* and miR159 and miR164 target two *LuCAMTA* genes each. The predicted miRNAs were reported to involve in cleaving and inhibition of the translation of target genes.

**Table 3:** miRNA targets of potential *CAMTA* genes in flax.

miRNA_Acc.	Target_Acc.	Expectation	UPE	Alignment	Inhibition	Multiplicity
lus-miRN30	LuCAMTA1	2.5	15.742	miRNA AAUGGAGAGUUCGGAAAGAAG	Translation	1
				Target UCUCUUUCCGUACUCUCCGUG		
lus-miRN9	LuCAMTA1	3.5	15.98	miRNA UUCUUUGGCUGAGAAUUGGAG	Cleavage	1
				Target UUCUGAUUAUCAGGCAGAGAA		
lus-miR2275	LuCAMTA2	4.5	16.74	miRNA UUUAGUUUCUUCCAAUAUCUUU	Cleavage	1
				Target AUGUAUGUUUGGAGAAGUUGAA		
lus-miR164	LuCAMTA3	4.5	22.151	miRNA UGGAGAAGCAGGGCACGUGCA	Cleavage	1
				Target UUCAUGCGUACUGCUUCGCCA		
lus-miR159	LuCAMTA4	4	15.24	miRNA UUGGGGUGAAGGGAGCUCCC	Cleavage	2
				Target UGUAGCUCACUUUAUUUCAA		
lus-miR164	LuCAMTA5	3.5	14.66	miRNA UGGAGAAGCAGGGCACGUGCA	Cleavage	1
				Target UUCACGUCUUCUGCUUCUUCU		
lus-miRN15	LuCAMTA5	4	17.571	miRNA UUGCUGACAGAUUAUUUCGGU	Translation	1
				Target UUUGGAAUUAGUUGUCAGUAA		
lus-miR395	LuCAMTA6	4	14.418	miRNA CUGAAGUGUUUGGAGGAACUC	Translation	1
				Target CGUUUCCUCUAACUGUUUCAG		
lus-miR156	LuCAMTA7	4.5	12.93	miRNA UGACAGAAGAGAGUGAGCAC	Translation	3
				Target CUUUUCAUUCGUGUCUGUCA		
lus-miRN28	LuCAMTA7	3.5	23.11	miRNA UUGAACUGUACUAGUUGUCUGA	Cleavage	1
				Target AAAGACA-CUUGUACAGUUCAG		
lus-miR164	LuCAMTA8	4	17.34	miRNA UGGAGAAGCAGGGCACGUGCA	Cleavage	2
				Target ACUAUGGGCCUUGAUUCUUCA		
lus-miR164	LuCAMTA9	4	17.409	miRNA UGGAGAAGCAGGGCACGUGCA	Cleavage	2
				Target ACUAUGGGCCUUGAUUCUUCA		

## Discussion

The divalent ion calcium ion (Ca^2+^) plays a key role as a core transducer and regulator in response to environmental stimuli and developmental processes of plants [1]. Ca^2+^ signals are decoded into appropriate physiological responses and transmitted to the sink [2, 3]. CaM is an important Ca^2+^-binding protein with a defined role in biochemistry, cell biology and molecular biology as a regulator that binds to a number of target proteins [2, 3, 72]. CAMTA transcription factors play pivotal roles in calcium/calmodulin transduction signaling pathways, and CAMTA-mediated gene transcription regulation, key processes for plants’ responses to exogenous hormones and abiotic stresses [33, 73–75]. The current study identified nine members of flax *CAMTA* gene family. A combined N-J tree was developed to establish a phylogenetic relationship between Arabidopsis and flax. The analysis revealed an intimate association between CAMTA transporters in Arabidopsis and flax, indicating that the roles of LuCAMTAs could be like those of AtCAMTAs (Fig 1). Interestingly, three genes of the *LuCAMTA* gene family (LuCAMTA1-3) from group- I exhibited a close association with three At*CAMTA genes* (AtCAMTA1-3). Reportedly, these genes have been well-investigated for their participation in SA-regulated defense response and tolerance to cold stress [33, 34]. The results show that LuCAMTA1, LuCAMTA2, and LuCAMTA3 are closely related and hence they may function together in a similar pathway as homolog genes. Four members of the group- III in flax (LuCAMTA6, 7, 8, and 9) were clustered with AtCAMTA6, which was reported for its role during salt stress and SA signaling [37], indicating the possible role of LuCAMTAs in this group under salinity stress and hormonal regulations.

The structure of all the genes of *LuCAMTA* family was analyzed to make a mutual comparison for their structural diversity. Intron number of these genes showed a variation from 9 to 12, with a little deviation in various groups. For instance, *CAMTA* genes of group III and I were disrupted by the highest numbers of introns i.e. 9–12, while group II was disrupted by 9–11 introns. The fixed number of introns and exons is a conserved character of CAMTAs, which is an inherited trait also demonstrated by CAMTA family of other species like Arabidopsis, maize and tomato [12]. Intron phases also show conserved nature along the same group and show variations among different groups.

Study of protein structure is important to understand its mode of action. The conserved motifs of flax CAMTAs protein were analyzed by using the MEME; Multiple Expectation Maximization for Motif Elicitation online database. The plant CAMTA-encoded proteins were characterized with the presence of four functional domains, known as CG-1 (a sequence-specific DNA-binding domain), ANK (ankyrin repeats), IPT/TIG (transcription factor immunoglobulin), and IQ motifs (calmodulin-binding) [24–27]. The major basic domains such as CG-1, ANK, IPT/TIG and IQ were found within the *LuCAMTA* gene family which, are highly conserved across the species [14, 17, 20, 76].

To elucidate the transcriptional regulation in response to stress and hormones, PlantCARE database was accessed. The *cis-* regulatory elements were predicted in the 1Kb upstream promotor region of *LuCAMTA*. The current study revealed four stress-responsive elements; low-temperature-responsive (LTR) elements [77], anaerobic induction (ARE) elements [78], drought responsive (MBS) elements [79], and light responsive (G-box) elements [80]. Promoter analysis also indicated Hormone-responsive elements like abscisic acid-responsive (ABRE) [81] and salicylic acid-responsive elements (TCA element) [82]. The presence of *cis-* regulatory elements, responsive to hormones and stress, in the promotor regions of *CAMTA* gene family reveals their role in corresponding environments.

GO annotation suggested three basic types of functional classification i.e. cellular structural component, CC; molecular functions, MF; and biological processes, BP [83]. The system is extensively used to determine the gene functions in different organisms. The proteins encoded by *LuCAMTA* genes were submitted to GO database to determine the functions of these genes. According to the results, *LuCAMTA* genes were involved in BP, MF and CC. Regarding cellular structural component (CC), LuCAMTAs were responsible for intracellular and cellular anatomical components. The genes regarding molecular functions (MF), carried out sequence-specific DNA binding activities, while the genes in biological processes (BP) were found to regulate the responses to stimuli, biological processes and metabolic processes (Fig 6).

MicroRNAs (miRNAs) are endogenous small RNA sequences of 20–24 nucleotides, performing pivotal functions in regulating growth and developmental processes of plants. They down-regulate the expression of their corresponding genes at post-transcription stage by gene silencing and target degradation or translational repression. To understand the regulatory mechanisms in plants, Identification of miRNAs is of supreme importance. Previous reports have revealed 32 conserved miRNAs in flax [84]. Plant small-RNA target (psRNATarget) analysis server was used to search the potential miRNA targets in a set of nine identified LuCAMTA transcripts. Predicted miRNAs were related to different miRNA families including miRN30, miRN9, miR2275, miR164, miR159, miR164, miRN15, miR395, miR156, miRN28, miR164. These miRNAs have definite roles in different biotic and abiotic stresses [85].

## Conclusion

The current study reports the first systematic analysis of *CAMTA* genes in flax (*Linum usitatissimum*). The members of *CAMTA* gene family in flax were identified and characterized by in silico approaches. Nine genes of CAMTA family were identified in flax genome. The analysis of these genes also suggested a potentially functional association with transporters of other plant species. The current study also identified different miRNA families targeting the identified genes of CAMTA family in flax. The present findings are of great importance to elucidate the involvement of *CAMTA* gene family in metabolic processes of flax and for identification of key genes in future breeding programs. The current analysis provides a deep insight into *LuCAMTA* gene family to enhance agronomic, ecological and economic benefits of flax.
